The article "Cellular Imaging Analysis Algorithm-Based Assessment and Prediction of Disease in Patients with Acute Lung Injury" was retracted in 2023. Reasons: signs of a paper mill; suspected computer-generated content; unreliable results or conclusions; concerns about the data.

# Cellular Imaging Analysis Algorithm-Based Assessment and Prediction of Disease in Patients with Acute Lung Injury

**DOI:** 10.1155/2022/3193671

**Published:** 2022-08-22

**Authors:** Liang Gao, Chengwang Xiao, Taoyi Cheng, Zhaohan Wang, Wenhan Xia

**Affiliations:** ^1^Department of Urology, Jiangxi Provincial People's Hospital, The First Affiliated Hospital of Nanchang Medical College, Nanchang 330000, China; ^2^The Third Department of Internal Medicine, Wannian Hospital of Traditional Chinese Medicine, Shangrao 335500, China; ^3^Department of Critical Medicine, Wannian Hospital of Traditional Chinese Medicine, Shangrao 335500, China; ^4^Department of Gastroenterology, Jiangxi Provincial People's Hospital, The First Affiliated Hospital of Nanchang Medical College, Nanchang 330000, China; ^5^Department of Critical Medicine, Jiangxi Provincial People's Hospital, The First Affiliated Hospital of Nanchang Medical College, Nanchang 330000, China

## Abstract

This paper uses cellular imaging analysis algorithms to assess and predict the condition of patients with acute lung injury. Given the unique optical properties of UCNPs, this paper designs a ratiometric upconversion fluorescent nanoprobe for the determination of nitric oxide (NO) content in living cells and tissues. To address the image degradation phenomenon of optical sections, this paper uses a blind deconvolution method to abate the degradation effect caused by the scattered focus surface, thus completing the image recovery. After that, grayscale and binarization are performed using the weighted average method and the Otsu method. In this paper, we propose a migration learning-based Resnet-50 network for the triple classification of unlabeled leukocytes based on the characteristics of cell images acquired by a miniaturized label-free microfluidic cell imaging detection device. The migration learning can rapidly optimize the network parameters, the short connection structure of Resnet-50 is more suitable for feature extraction of unlabeled leukocytes than the InceptionV3 model without a short connection structure, and the accuracy of the Resnet-50 network can reach 94% in the test set. In this paper, we propose two tracking algorithms based on the dynamic Gaussian mixture model and mathematical morphology-based algorithms suitable for cells of different shapes for cell tracking in microscopic images, neuronal cell labeling in fluorescent images, and cell segmentation in mice. These methods have the advantages of low cost, speed, reproducibility, and objectivity, and we hope that their elicitation will be useful for relevant cell biology research.

## 1. Introduction

Acute lung injury (ALI) is inflammation and increased permeability of the lung caused by various pathogenic factors inside and outside the lung other than the cardiac origin, and multiple injuries are one of the main causes of morbidity and mortality. Studies on the behavior of cell migration, deformation, division, and adhesion play an important role in biomedical fields such as embryonic development, parasite invasion, immune response, wound healing, and cancer [1]. While the abundance of imaging tools makes it easy to observe living cells, the image data generated also poses new challenges for analytical processing because the motion of individual cells is relatively random, and to obtain certain motion indicators, the results must be obtained by averaging many cells over a long period. For example, studying the cytoskeleton, which determines many aspects of cell morphology and motility, is regulated by a variety of proteins, and most changes in the cytoskeleton have very limited effects when they occur, which are difficult to detect without quantitative analysis but an only visual observation [2]. In other words, quantitative analysis is essential for the construction of cellular behavior models and thus for the understanding of cellular behavior patterns. With the maturation of Drosophila RNAi technology that interrupts gene expression and enables screening of the entire genome to study the effects of specific genes on cellular function, we aim to use image-based high-throughput RNAi screening to discover effectors of Rho proteins and ds RNA that causes Rho-induced loss of cytoskeletal structure to identify possible effectors. However, the total number of images acquired is several million, which is completely beyond the scope of manual analysis to tolerate, and arguably, automated analysis is the only feasible way to address this problem. Dexmedetomidine can significantly reduce the lung injury caused by LPS, while the inhibitor yohimbine can reverse the effect of dexmedetomidine on reducing lung injury, which further indicates that dexmedetomidine has the function of lung protection.

The article "Cellular Imaging Analysis Algorithm-Based Assessment and Prediction of Disease in Patients with Acute Lung Injury" was retracted in 2023. Reasons: signs of a paper mill; suspected computer-generated content; unreliable results or conclusions; concerns about the data.

There is no doubt about the efficacy of adjuvant therapy for cancer, especially with the development and application of new drugs in recent years. However, adjuvant therapy has brought new problems to the clinic while producing obvious efficacy; that is, it has increased side effects [3]. Firstly, the side effects of drug therapy include bone marrow suppression and liver and lung injury. Bone marrow suppression and liver injury are generally well-controlled at present, but with the continuous development of newer and more widely used antitumor drugs, the incidence of lung injury is also increasing. Secondly, radiation lung injury is one of the common adverse effects of cancer radiation therapy [4]. The lung injury caused by chemotherapy drugs or targeted antitumor drugs in adjuvant therapy is drug-induced (DILI), which is an adverse reaction to the respiratory system (including lung tissue, bronchi, pulmonary vessels, and pleura) caused by drug therapy and can lead to respiratory failure in severe cases. The clinical manifestations of DILI are nonspecific and mainly consist of chest pain, dyspnea, fever, cough, and, in severe cases, respiratory failure. Acute lung injury includes acute interstitial pneumonia, noncardiogenic pulmonary edema syndrome, ARDS, and pleurisy. Late lung injury occurs after 2 months of treatment, and imaging shows pulmonary fibrosis.

D-dimer (D-D) is one of the markers of fibrin after the reaction of the coagulation process by the corresponding fibrinolytic enzymes. After the formation of acute aortic dissection (AAD), many thrombi are formed under the intima of the middle layer of the aortic vessels, and the human body's self-fibrinolytic mechanism is activated, resulting in fibrinolysis in the pulmonary microvasculature [5]. Many tiny thrombi are formed, and under the condition of a certain amount of ventilation in the lung, the blood flow in the lung is less than usual due to the thrombus, and the balance of ventilation/blood flow in the patient is broken, which in turn promotes the occurrence and development of acute lung injury to a certain extent. Regarding the further development of acute lung injury in acute respiratory distress syndrome (ARDS), whose mortality rate is up to 40% or more, early prognosis and intervention of acute lung injury have a certain role in improving the long-term survival rate, quality of life, and physicians' treatment modalities and have a more obvious role in the formulation of treatment plans for clinicians. They have a more obvious role in the development of treatment plans for clinicians [6].

## 2. Related Works

The cell is the basic component of an organism, and its structure and function are important for life activities. Cells are not only containers for many chemicals but also complex systems consisting of membranes, vesicles, and signaling pathways. Understanding complex life processes requires the integration of information and knowledge from different levels [7]. In recent years, there have been popular and important advances in genomics, which provides tools for research at the gene level, and proteomics, which explores the structure, function, and interactions of proteins. While these results have provided new ways and means to understand the cell, they have also led to the realization that studies targeting genes and proteins alone are not sufficient in many cases and that continued in-depth exploration at the cellular level is necessary and urgent [8]. To diagnose and treat diseases through microscopic images, cellular images are becoming increasingly important in medical imaging and research of corresponding diseases. Cell images facilitate better observation of the morphology, optical density, and other image features of cells or cell structures, but the process of acquiring images requires cell culture, smear production, microscopic imaging, and other steps, making cell images characterized by strong noise, blurred images, and uneven images, which need to be combined with sophisticated image processing techniques to process the acquired cell images to obtain disease information and make an accurate diagnosis. In the process of processing cell images by computer systems, image segmentation, feature extraction, and classifier design are three key issues, and since the CLSM images used in this project only image individual cells, the impact of phenomena such as cell stacking on the accuracy of image segmentation and feature extraction is avoided [9]. As an automated medical aid diagnosis method, automatic analysis based on cell images can qualitatively and quantitatively identify the source and cause of disease efficiently and accurately. Automatic classification of cells using pattern recognition relies mainly on the feature parameters of cell images. When extracting cell features in general, most researchers mainly take morphological features, optical density features, and texture features. Xie et al. [10] proposed a polygon fitting-based algorithm for cell image features [10]. Braune et al. [11] extracted morphologically color features of lung cancer cells and used neural networks to achieve automatic recognition [11]. Wu et al. [12] extracted frequency features of cell images using Fourier transformation of images for cell classification. For automatic cell classification, several machine learning methods have been used for cell feature classification [12].

The article "Cellular Imaging Analysis Algorithm-Based Assessment and Prediction of Disease in Patients with Acute Lung Injury" was retracted in 2023. Reasons: signs of a paper mill; suspected computer-generated content; unreliable results or conclusions; concerns about the data.

Acute aortic coarctation occurs when the aortic intima produces a rupture and blood flow into the false lumen in contact with the extracellular matrix of the middle layer of the aorta leading to the activation of inflammatory cells and the release of a series of inflammatory factors such as interleukin-6 (IL-6), interleukin-8 (IL-8), tissue factor, and other related inflammatory factors, leading to extensive alveolar exudation in the patient's lung, resulting in interstitial edema and affecting the patient's pulmonary ventilation function, which leads to developing hypoxemia that is difficult to correct [13]. The central mechanism for the development of acute lung injury is the waterfall inflammatory response, and Sparks et al. [14] suggested that a “waterfall-like” response due to inflammatory factors is involved in the development of acute aortic coarctation [14]. Camiolo et al. [15] and Maher et al. [16] reported that C-reactive protein (CRP) is a predictor of uncorrectable hypoxia in patients with acute aortic coarctation, suggesting that the inflammatory response secondary to acute aortic coarctation is associated with decreased oxygenation [15, 16]. Another mechanism illustrated is the slow flow rate of blood into the false lumen, thrombosis, and secondary fibrinolytic hyperfunction, resulting in a hypercoagulable and hypofibrinolytic state of systemic blood, in which fibrin deposition in the pulmonary microvasculature and vasculature due to the hypercoagulable and hypofibrinolytic state of the blood is one of its characteristics.

The pathogenesis of ALI is a combination of several factors and has not yet been fully investigated. Acute lung injury is clinically manifested by progressive dyspnea, distress, and uncorrectable hypoxemia, mainly due to hypoxia. The pathology is mainly characterized by acute alveolar exudation, resulting in interstitial edema, extensive intrapulmonary microvascular endothelial damage, microthrombosis, and intra-alveolar fibrin deposition [17]. Without timely management and intervention, acute lung injury can progress further to acute respiratory distress syndrome. The latest foreign research findings now suggest that the lungs of patients may develop pulmonary fibrosis, leading to irreversible consequences and permanent lung failure; there are also some molecular cellular level studies suggesting a relationship between relevant signaling pathways and acute lung injury. These factors include disruption of coagulation, a “waterfall-like” inflammatory response, and several other factors that are not yet known and that deserve to be explored and studied in terms of materials and methods.

## 3. Cell Imaging Analysis Algorithm Design

Ultrasensitive detection of biochemical molecules is particularly important in the fields of food safety, clinical diagnosis, environmental monitoring, antibioterrorism, and biomedical research. In recent years, with the development of interfacial modification technology, nanotechnology, molecular assembly technology, and molecular recognition technology, modern optical detection technology has been widely used for the detection of biomolecules with its advantages of simplicity, convenience, and sensitivity [18]. Fluorescent probes have gradually become one of the powerful tools for molecular sensing and imaging due to their high sensitivity, high spatiotemporal resolution, and easy preparation. Usually, in a fluorescence sensing system, the information of the inducer can be known by analyzing the data. Conventional fluorescent probes generally consist of a recognition group (receptor), a reporter group (fluorophore), and a linker group (spacer). The recognition group identifies the analyte and determines the specificity of the analyte detection; the reporter group mainly shows the signal conversion, indicating that the analyte has been successfully captured, which determines the sensitivity of the probe; the linker group is used to connect the receptor and fluorophore to transmit the signal. When the analyte encounters the recognition group, it causes the fluorescence signal of the reporter group to change, and the purpose of detecting the analyte can be achieved by analyzing the data change. By retaining individuals with higher fitness, the approximate solution with the highest fitness is continuously evolved through operations such as crossover, mutation, and replication, and the code of the optimal individual in the last generation population is obtained, which can be regarded as the optimal solution of the problem.

The article "Cellular Imaging Analysis Algorithm-Based Assessment and Prediction of Disease in Patients with Acute Lung Injury" was retracted in 2023. Reasons: signs of a paper mill; suspected computer-generated content; unreliable results or conclusions; concerns about the data.

Five classes of features (histogram, grayscale cooccurrence matrix, grayscale gradient cooccurrence matrix, Gabor wavelet features, and shape size features) were extracted from each ADC image, for a total of 133 features. Also, interobserver variability of image histology extraction was assessed using intraclass correlation coefficients (ICC) with the following criteria: ICC < 0.50, poor agreement; 0.50 ≤ ICC < 0.70, moderate; 0.70 ≤ ICC < 0.80, good; ICC ≥ 0.80, excellent. The 133 imaging histology features were included in the feature screening algorithm along with 9 clinical and imaging features, here using the random forest for feature screening. The relative importance of each feature for predicting drug resistance was estimated using 500 decision trees in the training set to calculate the Gini index (Gini coefficient). The top 9 most relevant parameters were then filtered from these as model input parameters, and the details are shown in Figure 1.

This operation effectively avoids the instability of the three-dimensional posture and position of the cells caused by the experimental operation and CLSM shooting and ensures the stability and repeatability of the two-dimensional features of the image. To enhance the quality of cell images acquired by small portable devices and facilitate cell image detection, this paper uses the parallel residual super-resolution network PRSRCN for super-resolution processing of low-pixel cell images. Compared with the classification network, the super-resolution network replaces the classification layer with the reconstruction layer [19]. The super-resolution networks can be classified into two categories according to the input image: (1) the input image is the same size as the output image; (2) the input image is *N* times smaller than the output image (*N* is the magnification of the image). The image reconstruction layer of super-resolution networks will vary according to the input image size. For example, the most classical SRCNN network belongs to the first category of cases, while the ESPCN network belongs to the second category of cases. The algorithm diagram of the deep learning-based super-resolution network designed in this paper is shown in Figure 2.

The article "Cellular Imaging Analysis Algorithm-Based Assessment and Prediction of Disease in Patients with Acute Lung Injury" was retracted in 2023. Reasons: signs of a paper mill; suspected computer-generated content; unreliable results or conclusions; concerns about the data.

To compare different super-resolution algorithms (or models), it is common to use recognized super-resolution datasets for comparison (Set9, Set14, etc.). However, the judgment of the superiority of super-resolution recovery has always been an open issue, and it is inaccurate and unscientific to evaluate it with human eyes, so it is important to have a uniform evaluation standard.

(1) $$\begin{array}{c} MSE=\sum_{i=0}^{N}M+\sum_{j=0}^{N}n+1. \end{array}$$

The three-dimensional structure of cells was reconstructed by using the moving cube algorithm for face mapping of three-dimensional cell contours based on binarized images. However, due to the limitations of biological experimental operations and confocal microscope shooting angles, the 3D structures reconstructed by D-D optical sectioning have various poses and positions, which affect the consistency, accuracy, and stability of cell feature extraction and classification. Therefore, the method of finding the spatial long axis in the 3D contour is proposed, and the maximum profile obtained from the spatial long axis based on reslicing using the coordinate axis rotation method is used as the reference plane for feature extraction. Based on this, morphological features of the cell images are calculated, and feature analysis and selection are performed using genetic algorithms. Based on the selected features, the support vector machine with different kernel functions and multilayer perceptron with different network structures are used for classification and identification, the effectiveness of the algorithm is verified, the performance of classifiers with different structures is compared, and the recognition accuracy is up to 97.8%.

(2) $$\begin{array}{c} \text{Recall}=\frac{FN}{TP+FP}. \end{array}$$

The world coordinate system is the absolute coordinate system of the system. When the coordinate system with D-D as the user is not established, the coordinates of all points in the data set of each instance of D-D are used to determine the position of each point with the origin of the world coordinate system. The obtained 3D profile of the cell is a collection of points existing in the world coordinate system. The spatial long axis of the cell is the two points on the cell surface contour that are farthest apart. Let the coordinates of the points on the cell surface contour be (*x*_*i*_, *y*_*i*_, *z*_*i*_), *i*=1,2,…, *n*, where *n* is the total number of contour points. To calculate the spatial long axis, traverse the distance between all two points on the surface contour, and take the maximum value of which is the spatial long axis *d*_max_ of D-D, calculated as (2), where *i* ≠ *j* and *i*, *j*=1,2,…, *n*.

(3) $$\begin{array}{c} d_{\max}=\max\left({\sqrt{\left(x_{i}+x_{j}\right)+\left(y_{i}+y_{j}\right)}}^{2}+\sqrt{{\left(z_{i}+z_{j}\right)}^{2}}\right.. \end{array}$$

The genetic algorithm (GA) is a randomized search method that evolved from Darwinian evolution. It draws on the natural selection mechanism of survival of the fittest and combines with the genetic mechanism to obtain the code of the best individual in the last generation population by retaining the individuals with higher fitness and continuously evolving the approximate solution with the highest fitness through crossover, mutation, and replication operations, which can be regarded as the optimal solution of the problem. The 18 morphological features obtained are normalized using the designed normalization algorithm, and then the genetic algorithm is used for feature analysis and selection. The selection of D-D features was performed using a genetic algorithm. The separable criterion of intra- and interclass distance (Euclidean distance between features) was used as an adaptation function. The number of D-D morphological features was 20. The population size was 8, the probability of fixing the occurrence of the crossover was 0.5, and a limit was placed on the number of iterations (100). A genetic algorithm is executed 15 times for feature selection for D-D cell classification, and the feature is selected as the target feature when the binarization of the feature parameter has a value of 1 more than 9 times. After selection, a total of 9 features were selected. The selected features are cytoplasmic maximum profile area Ac, cytoplasmic maximum profile perimeter Pc, cytoplasmic maximum profile roundness Cc, cytoplasmic maximum profile elongation Ec, cytoplasmic maximum profile roughness RAc, cytoplasmic maximum profile fractal dimension DIMc, eccentricity T, and stereospecific nucleoplasmic ratio NP.

(4) $$\begin{array}{c} y_{i}=\left[\left(w^{T}x_{i}\right)-b\right]+1,i=1,2,\ldots ,n. \end{array}$$

The article "Cellular Imaging Analysis Algorithm-Based Assessment and Prediction of Disease in Patients with Acute Lung Injury" was retracted in 2023. Reasons: signs of a paper mill; suspected computer-generated content; unreliable results or conclusions; concerns about the data.

## 4. Acute Lung Injury Modeling

The procedures for the construction of a mouse model of acute lung injury are as follows:

(1) Experimental animal selection:all mice were housed at an appropriate temperature and humidity in a 12 : 12-hour light and dark cycle environment, with free access to standard food and water. All animal experiments were approved by the ethics committee of the University of Medicine and were conducted following the principles of the university's laboratory guidelines.
(2) Anesthesia and fixation of animals: mice were anesthetized with 2.5% aphrodisiac (10 *μ*l/g) by volumetric intraperitoneal injection, and the neck of mice was prepared for skinning. Then the mice were placed supine on the bubble plate, the limbs were straightened and fixed with medical tape, the mice's head was tilted back, and the incisors were hung on the bubble plate with thick wires.
(3) Exposure of trachea: the skin of the neck was disinfected by wiping with iodine volts, and the trachea was exposed by cutting the skin 1.5 ∼ 2 cm along the midline of the neck and pulling apart the muscles and neck tissues.
(4) Intratracheal drip: the fixed mouse bubble plate was lifted to about 80° to the ground, with a good LPS work 1 ml syringe and the mouse trachea in a parallel direction into the mouse trachea 3 ∼ 4 mm, slowly advance the syringe, and drip drug syringe should be left for 5 s before pulling out. After pulling out the needle and then fixing the mouse bubble Mu plate and stay 10 s, and finally, suture the mouse neck skin.
(5) Twelve mice were randomly divided into 2 groups of 6 mice each.
  - Control group (control group, 6 animals): equal amount of saline was dripped into the trachea.
  - Polysaccharide group (LPS group, 6 animals): intratracheal drops of LPS 10 mg/kg were used to establish the animal model.
(6) After the two groups of mice were treated, the general status of the mice was observed in terms of activity, feeding condition, mental condition, and respiratory rate to determine whether the sepsis lung injury model was successfully constructed.

## 5. Algorithm Model Construction for Assessing and Predicting the Condition of Patients with Acute Lung Injury

The central mechanism of ALI is the formation of aortic coarctation, endothelial cell leakage, tissue factor release, and blood contact with the aortic intima, resulting in the release of histogenic factors, activation of cells associated with the inflammatory response, and the entry of a large number of inflammation-related factors into the blood, such as interleukin-6 (IL-6), interleukin-8 (IL-8), and other proinflammatory factors, resulting in a “waterfall.” This results in a “waterfall-like” inflammatory cascade, leading to extensive alveolar exudation and interstitial edema. Another more accepted mechanism is that blood entering the false lumen activates the coagulation system and forms a wall clot, which leads to a slow flow rate and thrombus formation due to reduced pressure in the aortic false lumen, secondary to activation of the fibrinolytic system and disruption of the systemic coagulation balance [20]. The lung is the tissue organ that receives all the cardiac output in the human circulation and is also the oxygenation system for the systemic venous blood flow, the high coagulation and low fibrinolytic state in the systemic circulation leads to the deposition of fibrin in the pulmonary microvessels and the vasculature, resulting in the formation of thrombus in the pulmonary microvessels, and the formation of microthrombus in the lung leads to the disruption of the balanced state of the pulmonary ventilation/blood flow ratio [21].

The article "Cellular Imaging Analysis Algorithm-Based Assessment and Prediction of Disease in Patients with Acute Lung Injury" was retracted in 2023. Reasons: signs of a paper mill; suspected computer-generated content; unreliable results or conclusions; concerns about the data.

To ensure the reliability of the results of subsequent bioinformatics analyses, we analyzed the processed dataset data with the Network Analyst online quality assessment tool using gene count plots, box line plots, density plots, and principal component analysis plots, respectively. The gene count plot (count sum) was used to calculate the number of genes in each sample. The box plot is used to show the normalization of data between microarrays, and the common method is median normalization. A density plot (plot of density) is a nonparametric method used to estimate the probability density function of a random variable and is an effective method used to observe the distribution of continuous variables. Principal Component Analysis (PCA) is one of the most widely used algorithms for dimensionality reduction of data. Its main purpose is to “reduce the dimensionality” by analyzing the largest individual differences in the principal components to find features that are easier to understand. Adjuvant therapy not only produces obvious curative effects but also brings new problems to the clinic; that is, it has more side effects. The side effects of drug therapy include bone marrow suppression and liver and lung damage.

In the D-D classification test, normal cells marked as 1 were considered positive cases, and senescent cells marked as 0 were considered negative cases. Based on the above four cases, True Positive Rate (TPR) and False Positive Rate (FPR) can be calculated, respectively. Taking the SVM classifier with polynomial kernel function as an example, the 8th sample is obtained using random sampling, each group contains 100 practice samples (including 59 normal cells and 41 senescent cells) and 45 cases as test samples (including 28 normal cells and 17 senescent cells), and the confusion matrix of binary classification is calculated with the ROC curve after classification. For the ROC curve, the closer to the upper left corner of the model, the higher the classification accuracy, and the area under curve AUC (Area under Curve) = 0.921 was obtained by calculation. The ROC curve of D-D classification is shown in Figure 3.

The article "Cellular Imaging Analysis Algorithm-Based Assessment and Prediction of Disease in Patients with Acute Lung Injury" was retracted in 2023. Reasons: signs of a paper mill; suspected computer-generated content; unreliable results or conclusions; concerns about the data.

As an activation function, the full input weighted summation is entered into it. Thus, the activation function completes the mapping between the input and output. The activation function gets its name from its function: activating the corresponding neuron to get the corresponding output.

(5) $$\begin{array}{c} \text{sigmoid}\left(x\right)=1+\frac{1}{1-e^{x}}. \end{array}$$

The Sigmoid function has a monotonically increasing output value of (0, 1) and a smooth output. However, the output is not 0-centered and has soft saturation, and *x*_1_ is susceptible to gradient dispersion, which leads to deactivation of neurons during training.

The normalized exponential function (Softmax) function is commonly used in the output of a multiclassification neural network, which can normalize the reliability of each category of classification to the form of a probability that the sum of the classifications is 1. The functional form is

(6) $$\begin{array}{c} \text{softmax}\left(x\right)=\sum_{k=1}^{k}e^{z_{k}}. \end{array}$$

The parallel residual superresolution network was trained in the Tensorflow framework using Python 2.7. The initial learning rate is set to 0.001, and the learning decreases to 0.5 times the initial learning rate every 9 epochs (24000 data trained in each epoch) until the learning rate decays to 10–5. The use of learning rate decay avoids problems such as slowing down the training speed or excessive oscillation of the lost value due to the consistently high learning rate. The stochastic gradient descent algorithm is used for updating the weight values, and the optimization method of adaptive moment estimation (Adma) is added to it. Stochastic gradient descent can speed up the training speed, and the adaptive moment estimation algorithm can optimize the first-order gradient of the objective function, which is more effective for large-scale parameter optimization.

(7) $$\begin{array}{c} \text{softmax}\left(x\right)=\sum_{k=1}^{k}e^{z_{k}}. \end{array}$$

## 6. Results and Discussion

### 6.1. Cell Imaging Analysis Algorithm Results

MCF-7 cells were cultured with high-sugar DMEM, 10% fetal bovine serum (GIBCO), and 1% penicillin-streptomycin (10,000 U/mL, 10,000 *μ*g mL^−1^, Invitrogen). The cell culture incubator was maintained at a constant temperature of 37°C and a 5% CO_2_ level. The killing effect of different concentrations of UCNP@DMI-mSiO2@CD on MCF-7 cells after 48 h incubation was investigated by MTT colorimetric assay. In the cell uptake experiment, MCF-7 cells were incubated with UCNP@DMI-mSiO2@CD nanoprobe for 0.5 h, 1 h, 2 h, 3 h, and 4 h, followed by three washes with PBS, and then two-photon confocal imaging was performed with an excitation wavelength of 920 nm, a pulse width of 120 fs, and a repetition frequency of 80 MHz. z-axis scanning two-photon confocal imaging maps of MCF-7 cells were scanned at 2 *μ*m intervals. Before cell colocalization imaging experiments, cells were coincubated with UCNP@DMI-mSiO2@CD for 2.5 h, followed by the addition of LysoTracker® Blue DND (1.0 *μ*Μ) for 30 min, and finally washed three times with PBS. Nigericin is a standard method for regulating the *pH* consistency within cells and cell cultures and can be used for intracellular *pH* calibration experiments. Therefore, cells were incubated with UCNP@DMI-mSiO2@CD nanoprobes for 2.5 h and then incubated with different *pH* KCl buffers (10 *μ*M nigericin, 120 mM KCl, 1 mM CaCl_2_, 30 mM NaCl, 1 mM NaH_2_PO_4_, 5 mM glucose, 0.5 mM MgSO_4_, and 20 mM HEPES) for 30 min.

The article "Cellular Imaging Analysis Algorithm-Based Assessment and Prediction of Disease in Patients with Acute Lung Injury" was retracted in 2023. Reasons: signs of a paper mill; suspected computer-generated content; unreliable results or conclusions; concerns about the data.

So, we focus on how to label all the neurites. For many cellular tests, biologists tend to be more concerned with the statistical regularities of neuronal structure, rather than individual neurons. Unlike previously proposed semiautomatic neuron labeling methods, our goal is to design a fully automatic labeling algorithm that can label all neurons in a graph simultaneously without human manual intervention and at most requires setting fewer parameters. Because our method is automatic and the difference between automatic and manual labeling results is small, manual intervention is not required for practical labeling applications, especially for large numbers of images. However, manual modifications can sometimes be helpful to ensure user satisfaction, so we also record the amount of work spent on the inspection process to have a quantitative idea of the number of manual modifications that may be required [22]. We consider here two quantities, which are the number of modified positions and the cumulative modification time (in seconds), and for both observers, the box plots of these two quantities are shown in Figure 4, where the mean and variance of the number of modified positions are 3.3273 and 2.0463 for observer 1 and 3.3636 and 2.0938 for observer 2, and the mean and variance of the cumulative modification time for observer 1 are 10.1636 and 6.3239 for observer 1 and 10.0909 and 6.2754 for observer 2; it can be seen that, in general, only fewer modifications are needed to satisfy the observers.

The article "Cellular Imaging Analysis Algorithm-Based Assessment and Prediction of Disease in Patients with Acute Lung Injury" was retracted in 2023. Reasons: signs of a paper mill; suspected computer-generated content; unreliable results or conclusions; concerns about the data.

The spatial long axis was calculated by using the 3D cell profile, and the reslicing of the 3D cell structure was realized by using the coordinate axis rotation method based on the spatial long axis to calculate the maximum cell profile as the reference plane for feature calculation, which effectively avoided the immobility of the 3D cell pose and position caused by the experimental operation and CLSM shooting, and ensured the stability and repeatability of the 2D features of the image [23]. Based on the selected cell features, support vector machines with different kernel functions and multilayer perceptrons with different network implicit layers were constructed to verify the algorithm city by classifying and recognizing the dataset and comparing the effects of different structural machine learning models on classification recognition to determine the best classification model. To prevent the transition of model fitting, the designer in this paper performs data augmentation on the 128 samples obtained and selects the Keras function for data augmentation. The modules in Keras can realize basic data augmentation functions (Figure 5).

For the cell images, the PSNR and SSIM values of the SRCNN model are significantly lower than those of the other four models, indicating that the super-resolution ability of the SRCNN model is inferior to the other four models, which may be caused by the fact that the SRCNN model is too simple to fully capture the eigenvalues of the cell images. Comparing the PSNR and SSIM values of the training model with different downsampling multiples of 1220 datasets and 305 datasets, we can see that the model recovery can be high in some cases using the dataset enhancement method. The PSNR and SSIM values of the training model with different downsampling multiples of 1220 datasets and 305 datasets show that the use of dataset augmentation can have a high model recovery effect in some cases.

### 6.2. Simulation Experiments of the Algorithm Model for Assessing and Predicting the Condition of Patients with Acute Lung Injury

In the control group, mice moved freely, breathed steadily, and did not see any abnormal diet; in the LPS group, mice showed behavioral changes such as restlessness, shortness of breath, poor mental status, and not thinking about eating and drinking after 30 minutes of intratracheal LPS drip, and a few mice had pink foam-like liquid flowing out around the mouth and nose. The behavioral results suggest that our model of acute lung injury established by intratracheal LPS drip was successful. The clinical manifestations of DILI are mostly nonspecific, mainly chest pain, dyspnea, fever and cough, and respiratory failure in severe cases.

The article "Cellular Imaging Analysis Algorithm-Based Assessment and Prediction of Disease in Patients with Acute Lung Injury" was retracted in 2023. Reasons: signs of a paper mill; suspected computer-generated content; unreliable results or conclusions; concerns about the data.

The wet-to-dry weight ratio (W/D) of lung tissue was used to evaluate the degree of edema of lung tissue, and the results showed that the W/D of the control group was 3.55 + 0.48, the WD of lung tissue of the LPS group was 8.9010.32, the W/D of the LPS + DEX group was 5.20 Earth 0.55, and the WD of the LPS + DEX + Yoh group was 8.31sh 0.45. Compared with the LPS group, the W/D of the LPS + DEX group decreased, and the difference was statistically significant, *P* < 0.05, while the WD of the LPS + DEX + Yoh group also decreased, but the difference was not statistically significant, *P* > 0.05. The results indicated that dexmedetomidine significantly reduced the pulmonary edema caused by LPS, while yohimbine, an inhibitor of *a*2-adrenoceptors, reversed the effect of dexmedetomidine in reducing pulmonary edema caused by LPS, as shown in Figure 6.

To evaluate the degree of lung injury, HE-stained pictures were scored, and the results showed 2 + 0.81 in the control group, 8 + 0.81 in the LPS group, 410.75 in the LPS + DEX group, and 7 out of 0.81 in the LPS + DEX + Yoh group; compared with the control group, the lung injury scores in the other three groups were increased, and the difference was statistically significant, *P* < 0.05. Compared with the LPS + DEX group, the lung injury score in the LPS + DEX + Yoh group increased significantly, and the difference was statistically significant, *P* < 0.05 compared with the LPS + DEX group. The difference was statistically significant, *P* < 0.05. The results indicated that dexmedetomidine significantly reduced the lung injury caused by LPS, while the inhibitor yohimbine reversed the effect of dexmedetomidine in reducing lung injury, which further indicated the lung-protective function of dexmedetomidine, as shown in Figure 7.

In addition, we further evaluated the effect of dexmedetomidine on acute lung injury by HE staining of lung tissues and pathological scoring of lung injury. The results of HE staining of lung tissues showed that the alveolar and other structures of lung tissues in the control group were intact, with no hemorrhage and no inflammatory cell infiltration; the LPS group showed severe alveolar structural damage, with many inflammatory cells infiltrating around the bronchi and in the alveoli, and obvious interstitial edema and congestion and hemorrhage in lung tissues; the LPS + DEX group showed slight alveolar structural damage. Compared with the control group, the lung injury scores in the other three groups were higher, and the difference was statistically significant, *P* < 0.05. DEX group lung injury score decreased, and the difference was statistically significant, *P* < 0.05, while the lung injury score in the LPS + DEX + Yoh group also decreased, but the difference was not statistically significant, *P* > 0.05; compared with the LPS + DEX group, the lung injury score in the LPS + DEX + Yoh group was significantly higher, and the difference was statistically significant *P* < 0.05 compared with the two groups. The results suggest that dexmedetomidine can significantly reduce the lung injury caused by LPS, while yohimbine, an inhibitor of *α*2-adrenoceptors, can reverse the effect of dexmedetomidine in reducing the lung injury caused by LPS.

The article "Cellular Imaging Analysis Algorithm-Based Assessment and Prediction of Disease in Patients with Acute Lung Injury" was retracted in 2023. Reasons: signs of a paper mill; suspected computer-generated content; unreliable results or conclusions; concerns about the data.

The mean values of the obtained CT image parameters of the positive group, as well as the grayscale values of the five percentile (including Perc01%, Perc10%, Perc50%, Per90%, and Perc99%) and the independent samples *t*-test, were used to statistically analyze each image parameter of grade 1 and 2 lung injury; according to the results, the significance of all parameter values was less than 0.001, which was statistically significant. The CTCAE5.0 standardized grading of the corresponding CT indicators of each parameter had significant differences, as shown in Table 1.

### 6.3. Discussion

Acute lung injury is an acute hypoxic respiratory insufficiency caused by damage to the alveolar-capillary barrier caused by various pathogenic factors, resulting in diffuse interstitial and alveolar pulmonary edema. Many factors contribute to acute lung injury, including physical, chemical, and biological factors. This study is a simulation study and evaluation of acute lung injury induced by biological factors, that is, LPS, which is difficult to shed from the cell wall and which is shed by lysing and destroying cells when bacteria die and so on and exerts its toxicity by acting on animal cells and so on. It is also called endotoxin because it is not a toxin secreted outside the body by bacteria (exotoxin). In this study, the tracheal drip LPS was used for modeling. The local inflammatory response in the lung is more pronounced when the tracheal drip LPS is used for modeling, and the successful modeling time is shorter, which can avoid the influence of other interfering factors on the results of the experiment. The warehouse stores and analyzes DNA microarray chips and the *R* software package for analyzing genome chip data, which is beneficial for researchers to efficiently process and analyze biological information detected by microarray chips, obtain meaningful molecular information, and provide theories for disease-related research basis. Our results showed that the mice in the control group moved freely, breathed smoothly, and did not show any abnormalities in their diet; the mice in the LPS group showed behavioral changes such as restlessness, shortness of breath, poor mental status, and not thinking about eating and drinking after the LPS intratracheal drip, which indicated that the acute lung injury model could be successfully constructed by dripping LPS from the trachea. It provided the necessary prerequisites for the smooth conduct of the later experiments. However, this study is a single-center study with a small sample size, and it would be a great blessing for patients as well as a society if more observational indicators could be detected later through a multicenter and large sample study and if a rapid and accurate judgment could be made for timely intervention in patients with acute lung injury. Therefore, the causative factors, diagnostic criteria, and therapeutic measures of ALI still need to be investigated, and further research on the molecular mechanism of its pathogenesis will be beneficial to the diagnosis and treatment of the disease and improve the prognosis of patients.

The article "Cellular Imaging Analysis Algorithm-Based Assessment and Prediction of Disease in Patients with Acute Lung Injury" was retracted in 2023. Reasons: signs of a paper mill; suspected computer-generated content; unreliable results or conclusions; concerns about the data.

## 7. Conclusion

This paper constructs a model for the assessment and prediction of the condition of patients with acute lung injury based on a cellular imaging analysis algorithm. This paper converts imaging data into objective values. Compared with previous studies, this study uses parameters at the largest level of the lesion extent instead of the entire whole lesion, thus providing a more accurate and easy diagnosis of the occurrence of lung injury while incorporating clinical factors of patients to study their risk factors for lung injury and providing a more objective diagnosis and grading method to assist in the treatment of related lung injury. The spatial long axis was calculated by using the 3D cell profile, and the reslicing of the 3D cell structure was realized by using the coordinate axis rotation method based on the spatial long axis to calculate the maximum cell profile as the reference plane for feature calculation, which effectively avoids the immobility of the 3D pose and position of cells caused by experimental operations and CLSM filming and ensures the stability and repeatability of the 2D features of the images. However, the number of cells that can be tracked by dynamic Gaussian mixture model-based cell tracking is relatively limited, generally, a few or tens, and the shape must be elliptical, which limits its application scope. And the mathematical morphology-based cell tracking assumes that there are obvious light and dark variations in various places inside the cells, which sometimes does not hold in practice and leads to its failure. It is hoped that more applicable tracking algorithms can be identified in the future.

The article "Cellular Imaging Analysis Algorithm-Based Assessment and Prediction of Disease in Patients with Acute Lung Injury" was retracted in 2023. Reasons: signs of a paper mill; suspected computer-generated content; unreliable results or conclusions; concerns about the data.

## Figures and Tables

**Figure 1:** Importance ranking of the 9 most relevant parameters.

**Figure 2:** Schematic diagram of super-resolution network algorithm.

**Figure 3:** ROC curve of D-D classification.

**Figure 4:** Box plot of the number of positions in the test and the cumulative modification time.

**Figure 5:** Learning curve of model classification recognition BMSCs.

**Figure 6:** Predicted wet-to-dry weight ratio of lung tissue.

**Figure 7:** Lung injury score.

**Table 1:** Image parameters of lung injury for independent sample prediction results.

Percent (%)	*F*	*P*	T	*P*
1	0.801	0.53	4.98	<0.001
10	0.621	0.903	4.77	<0.001
50	0.957	0.919	7.02	<0.001
90	0.579	0.738	7.38	<0.001
99	0.694	0.531	5.75	<0.001

## Data Availability

The data used to support the findings of this study are available from the corresponding author upon request.
